# Relationship between the UPLC Fingerprints of *Citrus reticulata* “Chachi” Leaves and Their Antioxidant Activities

**DOI:** 10.1155/2022/5834525

**Published:** 2022-11-22

**Authors:** Qin-Xin Nie, Qiu-Xia Zhang, Yin-Ji Zhu, Pei-Jun Wu, Ya-Li He, Jin-Yu Wang

**Affiliations:** ^1^School of Pharmaceutical Sciences, Guangzhou University of Chinese Medicine, Guangzhou 510006, China; ^2^Bioland Laboratory, Guangzhou 510700, China; ^3^Guangdong Yunfu Vocational College of Chinese Medicine, Yunfu 527499, China

## Abstract

*Citrus reticulata* “Chachi” (CRC) leaves contain abundant flavonoids, indicating that they possess good nutritional/pharmacological research and development potential. This study aims to explore chemical antioxidant quality markers based on the spectrum-effect relationship and quality control strategy of CRC leaves. The ultrahigh performance liquid chromatography (UPLC) system was used to establish chromatographic fingerprints of *Citrus reticulata* “Chachi” leaves. Simultaneously, they were evaluated by using similarity analysis (SA), hierarchical cluster analysis (HCA), and principal component analysis (PCA). Afterwards, the DPPH assay was adopted to study the antioxidant effects. The spectrum-effect relationship between UPLC fingerprints and DPPH radical-scavenging activities was studied with grey relational analysis (GRA). Analysis results indicated that there were twenty-one common peaks of fourteen batches of CRC leaves which were from different regions of Guangdong province, and their similarities ranged from 0.648 to 0.997. HCA results showed that fourteen batches of samples of CRC leaves could be divided into six classes at Euclidean distance of 5. The results from GRA showed that tangeretin and hesperidin were the main flavonoids responsible for the antioxidant activity in CRC leaves. In conclusion, this research established a chromatographic analysis method suitable for CRC leaves and demonstrated that chromatographic fingerprints analysis combined with the antioxidant activity could be used to evaluate the material basis of CRC leaves and may provide a reference to establish a quality standard.

## 1. Introduction

*Citrus reticulata* “Chachi” (CRC) is a citrus plant of Rutaceae family and can be used as medicine and food. At present, the application of CRC is mainly in the peel which is the source of citri reticulatae pericarpium (CRP) in Guangdong. CRP is used to treat respiratory and digestive system disorders including dyspepsia,acid reflux, constipation, and diarrhea, as well as the symptoms of other gastrointestinal diseases [1]. In order to protect and promote fruit, the leaves of CRC are regularly pruned every year, resulting in a large number of CRC leaves getting abandoned, which is a potential waste of resources. Only a small proportion of these leaves are used as foodstuffs, e.g., for tea making and spices. Preliminary studies by our research group found that the leaves of CRC also contained abundant flavonoids [2], indicating that they possess good nutritional/pharmacological research and development potential.

In order to expand the market application for CRC leaves, it is necessary to establish the quality control strategy and investigate the pharmacological efficacy. Therefore, this study aims to establish ultraperformance liquid chromatography (UPLC) fingerprints of fourteen batches of CRC leaves and to determine the contents of hesperidin, nobiletin, tangeretin, and 5-demethylnobiletin in fourteen batches of samples. Simultaneously, they are evaluated using similarity analysis (SA), hierarchical cluster analysis (HCA), and principal component analysis (PCA). Afterwards, the DPPH assay was adopted to study the antioxidant effects. The spectrum-effect relationship between UPLC fingerprints and DPPH radical-scavenging activities were studied with grey relational analysis (GRA). The correlation coefficient between the common peaks and the chemical antioxidant activity can be used to explore the quality markers of CRC leaves.

## 2. Materials and Methods

### 2.1. Materials and Reagents

Fourteen batches of CRC leaves were collected from different areas of Guangdong province in China for analysis, and the detailed information is listed in Table 1. The leaves were dried (60°C), reduced to coarse homogeneous powders, and stored in sealed containers at ambient temperature until required. Samples were authenticated by Prof. Kang Chen (College of Chinese Medicine, Guangzhou University of Chinese Medicine, Guangzhou, China).

Four reference compounds (≥98% purity) such as hesperidin, tangeretin, nobiletin, and 5-demethylnobiletin were obtained from Guangzhou Institute of Drug Control (Guangzhou, China); L-ascorbic acid was purchased from Damao Chemical Reagent Factory (Tianjin, China); and DPPH (≥97% purity) was obtained from Tokyo Chemical Industry Co., Ltd. (Shanghai, China).

Chromatographic grade acetonitrile was purchased from Merk (Darmstadt, Germany); ultrapure water was prepared in-house (18.2 MΩ·cm; Sichuan Zhuoyue Water Treatment Equipment Co., ltd., Sichuan, China); ethanol and phosphoric acid (analytical grade) were purchased from Merk (Darmstadt, Germany) and Tianjin Kemiou Chemical Reagent Co., Ltd. (Tianjin, China), respectively.

### 2.2. UPLC Fingerprints

#### 2.2.1. Preparation of Sample Extracts

Homogeneous sample powder (1.0 g) was extracted with aqueous ethanol (15 mL of 50% solution w/w) in an ultrasonic water bath (100 W, 40 kHz) for 50 min at room temperature. Additional aqueous ethanol was added to compensate for the weight loss during extraction, mixed well and passed through a 0.22 *μ*m membrane filter (Merck Millipore, USA) prior to UPLC analysis.

#### 2.2.2. Preparation of Standard Solutions

Standard solutions of hesperidin (0.654 mg/mL), tangeretin (0.398 mg/mL), nobiletin (0.120 mg/mL), and 5-demethylnobiletin (0.206 mg/mL) were prepared by dissolution in methanol; a mixed standard solution was obtained by combining 0.5 mL of each standard solution.

#### 2.2.3. UPLC Analysis

UPLC analysis was carried out using an ACQUITY™ UPLC™ H-Class Plus system (Waters, Milford, MA, USA) and a photodiode array detector. Extracts (2.5 *μ*L) were separated on an ACQUITY UPLC BEH C_18_ column (1.7 *μ*m, 2.1 mm × 100 mm) maintained at 35°C, prior to detection at 330 nm. The mobile phase consisted of acetonitrile (A) and 0.2% phosphoric acid (v/v) in water (B) at a constant flow rate of 0.3 mL/min and using the following elution program: 0–22 min, 8% to 24% solvent A; 22–29 min, 24% to 40% solvent A; 29–34 min, 40% to 50% solvent A; 35–37 min, isocratic 50% solvent A; and 37–40 min, linear gradient from 50% to 8.0% solvent A.

### 2.3. Methodology Validation

#### 2.3.1. Calibration Linearity

Calibration curves were obtained for each flavonoid (hesperidin, tangeretin, nobiletin, and 5-demethylnobiletin) by plotting the peak area response for each flavonoid standard (ordinate) at each of six concentrations (abscissa); linearity was assessed from the least squares fit to the calibration data.

#### 2.3.2. Instrumental Precision

Instrumental precision was determined from replicate (six) injections of a single sample extract solution; the peak areas of each flavonoid were recorded, and the RSDs were calculated.

#### 2.3.3. Repeatability

Repeatability was assessed from replicate analyses (six) of CRC leaves from the same batch; the RSD of the peak areas for each flavonoid were calculated.

#### 2.3.4. Stability

The stability was evaluated by reinjecting the same sample extract solution (see 2.2.1) at 0, 2, 4, 6, 8, 12, and 24 h; the RSDs of the replicate chromatogram peak areas and retention times for each flavonoid were determined.

#### 2.3.5. Recovery Test

Six sample powders (1.0 g each) of known flavonoid contents were fortified with an appropriate amount of each flavonoid. Samples were analyzed (see 2.2.1 and 2.2.3) and the recovery of each added flavonoid calculated.

### 2.4. Similarity Analysis

Data from the UPLC analysis were processed using “Similarity Evaluation System for Chromatographic Fingerprint of Traditional Chinese Medicine” software version 2012 (SESCFTCM) recommended by the State Food and Drug Administration of China [3, 4]. A simulated chromatogram, representative of fourteen fingerprints, was generated automatically by the software using the median method. Similarities between the chromatographic data from each of the different batches of samples and the reference chromatogram were then calculated.

### 2.5. HCA

The areas of common UPLC peaks were defined as characteristics to classify fourteen samples using SPSS Statistics for Windows, Version 26.0 software (IBM Corp., Armonk, NY, USA) [5, 6]. The between-groups linkage method and square Euclidean distance were used to measure the closeness of areas of common peaks among different samples.

### 2.6. PCA

PCA was applied to observe the distribution of samples in multivariate dimensional space and explore the relations among the independent variables. Thus, the common peaks of fourteen samples were analyzed by PCA using SPSS Statistics for Windows, Version 26.0 software (IBM Corp., Armonk, NY, USA). A principal component (PC) loadings matrix was constructed using the 21 peaks common to fourteen samples. The loadings values of each PC were then divided by the arithmetic square root of the eigenvalues of each autonomous component to give the linear model equations. After substituting the normalized peak areas of the 21 common peaks into the linear model, a PC score was obtained for each batch of samples.

### 2.7. DPPH Radical-Scavenging Assay

A working solution of DPPH (25 mg in 250 mL ethanol) was prepared and stored in the dark. L-Ascorbic acid was chosen as positive control (20 mg in 10 mL 50% ethanol), and the above solution was diluted with 50% ethanol into different concentrations of test solution for the later experiment. Sample extracts were serially diluted by 6.25, 12.5, 25, 50, 100, 200, and 400 times.

The DPPH working solution (100 *μ*L) was mixed with the diluted sample extract (100 *μ*L) in a 96-well plate. After incubating for 30 minutes in the dark, the absorbance of the reaction solutions was measured at 517 nm. The negative control solution without antioxidants was prepared and determined as the same manner. The free radical-scavenging capacity was calculated as follows: free radical-scavenging capacity (%) = *A*0 − *A*1/*A*0 × 100%, where *A*_0_ is the absorbance of negative control solution without antioxidants, and *A*_1_ is the absorbance of sample solution which is a mixture of free radical working solution and sample solutions. The results were expressed as the half maximal inhibitory concentration (IC50; mg/mL) [7, 8].

### 2.8. GRA

Grey relation analysis is an analysis method that includes multifactor statistical analysis. It uses grey relation grade to describe the degree of correlation between the data. IC_50_ was defined as the reference sequence, and the areas of common peaks from the UPLC fingerprint were defined as the comparison sequences. Standardizing the peak area and IC50 values of each sample by using GRA, the absolute difference sequence, the correlation coefficient, and the correlation degree were obtained. Finally, the potential antioxidant active components were screened according to the correlation degree.

## 3. Results and Discussion

### 3.1. UPLC Fingerprints

#### 3.1.1. Method Validation

To obtain stable and reproducible UPLC fingerprints, the retention times and peak areas for all characteristic peaks were measured relative to a reference peak (hesperin). The regression equations of hesperin, tangeretin, nobiletin, and 5-demethylnobiletin (Table 2) all showed good linearity (*R*^2^ > 0.999). The RSDs for the precision, repeatability, stability, and recovery of the reference flavonoids did not exceed 3% (Table 3). The correlation coefficients between the fingerprints obtained by repeated injection of the same sample extract solution and the common pattern fingerprints obtained were >0.95.

#### 3.1.2. Similarity Analysis

The overlaid chromatograms for samples from each batch of CRC are shown in Figure 1, and 3D chromatogram showing UV absorbance spectra at 300 nm is shown in Figure 2. There were 21 major peaks in UPLC chromatograms of all samples. Among these, four peaks were identified as hesperidin (peak 17), nobiletin (peak 19), tangeretin (peak 20), and 5-demethylnobiletin (peak 21; Figure 3). To compensate for any drift in retention time and change in peak area response, peak 17 was assigned as the reference to calculate the relative retention times (RRT) and relative peak areas (RPA) of each characteristic peak (Tables 4 and 5).

The results of the similarity analysis using SESCFTCM are listed in Table 6. The similarity data indicated that fourteen batches of samples were all different but within a moderate and acceptable range. When the similarity threshold was set to 0.9, samples 8 and 10 were dissimilar.

### 3.2. Content of Flavonoids

Amounts of each reference flavonoid in samples from each batch of CRC (Table 7) were identified and quantified from their UV spectra (Figure 4) and the slope and intercept of the linear regression calibration equations, respectively. Amounts of hesperidin were significantly greater than the other flavonoids; tangeretin showed the lowest concentrations in samples.

### 3.3. Antioxidant Activity

The antioxidant activities of fourteen batches of samples were determined using the DPPH assay. The results showed that the DPPH clearance rate was not linear with the concentration. Therefore, the Probit method in SPSS 26.0 software was used for regression analysis to fit the corresponding equation Probit (*p*) = Intercept + Bx, and then the IC50 values (the concentration of the sample solution when Probit = 0.50) was obtained. The IC50 values (Table 8; Figure 5) showed that the clearance rates for each sample followed the order as follows: S14 > S7 > S1 > S13 > S5 > S2 > S6 > S12 > S3 > S9 > S4 > S10 > S8 > S11.

### 3.4. HCA

The interval of intergroup connection and square Euclidean distance were used to establish a dendrogram of HCA of fourteen samples, which is shown in Figure 6. The HCA results show that the samples were mainly clustered into four classes at Euclidean distance of 10 and six classes at Euclidean distance of 5.

According to Table 1, the results of the HCA are not significantly correlated with their geographical locations. For example, S5 and S7, S12 and S2 are from same location, but they are grouped in different clusters. Since the bases where we collected CRC leaves are relatively limited, HCA results did not show obvious regional characteristics. At present, the main breeding methods of *Citrus reticulata* “Chachi” are ring-branch and grafting, and the flavor of fruit cultivated in different ways is also different. Moreover, the suitability of soil physical and chemical properties is crucial to the growth and development of plants and the accumulation of secondary metabolites [9]. In summary, other factors such as grafting or not, rootstock varieties for grafting and soil environment may affect quality of CRC leaves. Therefore, it is necessary to expand the scope of sample collection and comprehensively consider the factors such as soil factors, types of rootstock, and so on in the further study of CRC leaves quality classification and identification.

### 3.5. PCA

The data of the 21 common peaks from fourteen samples was subjected to PCA (SPSS 26.0). For extraction of standard eigenvalue of more than 1, the cumulative contribution rate of the first three components was 92.94%, indicating that the three principal components (PC) could represent most of the fingerprint information about fourteen samples. As shown in Tables 9 and 10, the eigenvalue in PC1 reached 14.565 with the variance contribution rate of 69.358%, and the peaks with higher loading were peak 3, peak 7, peak 14, and peak 15, indicating that these four peaks mainly reflected the information of PC1. The eigenvalue in PC2 was 2.585 with the variance contribution rate of 12.308%, and the peaks with higher loading were peak 12, peak 20 (tangeretin), and peak 21 (5-demethylnobiletin), indicating that these four peaks mainly reflected the information of PC2. The eigenvalue in PC3 was 2.367 with the variance contribution rate of 11.269%, and the peaks with higher loading were peak 12, peak 13, and peak 19 (nobiletin), indicating that these four peaks mainly reflected the information of PC3. To further visualize the results, the data were imported into SIMCA software version 15.0 (Umetrics, Sweden) to obtain two-dimensional analysis plot (Figure 7). As shown in Figure 7, the samples were mainly clustered into six categories: S10, S6, S4, S13, S3; S7, S12, S14, S11; S8; S2; S9; and S1, S5. The results of PCA were consistent with HCA. Among the samples, S8 distributed over the circle had poor quality, which was considered as an abnormal value, and this result was consistent with “similarity analysis.”

### 3.6. GRA

#### 3.6.1. Fingerprint-Efficacy Relationship

The relationship between the 21 common peaks and the DPPH radical-scavenging activity was established using the GRA model. The results showed that the contribution of each chromatogram peak (X) to the DPPH radical-scavenging activity was in turn (by number): X6 > X14 > X7 > X13 > X16 > X20 > X17 > X9 > X19 > X10 > X18 > X21 > X11 > X15 > X8 > X12 > X3 > X1 > X5 > X4 > X2 (Table 11). The results of correlation analysis between the 21 common peaks and the antioxidant activity showed that peak 6, peak 14, peak 7, peak 13, peak 16, peak 20 (tangeretin), and peak 17 (hesperidin) were the major components related to the antioxidant efficacy of the samples, and the correlation coefficients of 21 common peaks were more than 0.6, indicating that the antioxidant activity of the CRC leaves was the result of multiple ingredients synergy.

#### 3.6.2. Dose-Effect Relationship

The relationship between the measured amounts of hesperin, tangeretin, nobiletin, and 5-demethylnobiletin in each sample and DPPH radical-scavenging activity was also determined using the GRA model. The results showed that the contents of four flavonoids were not proportional to the antioxidant activity. The average contents of peak 20 (tangeretin) and peak 21 (5-demethylnobiletin) were low, but they had high correlation coefficient with the antioxidant activity. On the contrary, the content of peak 17 (hesperidin) was the highest compared with other three components, but it had the lowest correlation coefficient with the antioxidant activity (Table 12).

According to the reports in the literature, polymethoxylated flavones are a class of highly methoxylated flavonoids peculiar to citrus plants [10], which have antioxidant [11] cardiovascular and cerebrovascular disease prevention and anti-inflammatory effects. In this study, 5-demethylnobiletin and tangeretin had high correlation coefficient with the antioxidant activity. Therefore, the content of 5-demethylnobiletin and tangeretin in the CRC leaves can be used as the indexes for establishing the quality control strategy.

## 4. Conclusions

In conclusion, this research established a chromatographic analysis method suitable for CRC leaves and obtained good chromatographic separation. The results of GRA demonstrated that chromatographic fingerprints analysis combines with antioxidant activity could be used to evaluate material basis of CRC leaves. 5-demethylnobiletin and tangeretin in the CRC leaves can be used as the indexes for establishing the quality control strategy.

## Figures and Tables

**Figure 1:** Superimposed chromatograms of 14 batches of CRC leaves.

**Figure 2:** 3D chromatogram showing UV absorbance spectra of 300 nm.

**Figure 3:** Control fingerprint of CRC leaves (peaks 17, 19, 20, and 21 are hesperidin, nobiletin, tangeretin, and 5-demethylnobiletin).

**Figure 4:** UV absorption spectra of the reference flavonoids: (a): hesperidin, (b): tangeretin, (c): Nobiletin, and (d): 5-demethylnobiletin.

**Figure 5:** DPPH free radical-scavenger activity of fourteen batches of CRC leaves samples.

**Figure 6:** HCA dendrogram of fourteen samples.

**Figure 7:** PCA scores plot for the twenty-one common chromatographic peaks obtained from each of fourteen samples.

**Table 1:** Fourteen batches of CRC leaves from different areas.

Sample no	Origins
S1	Cixi county, Guangdong province
S2	Chakeng county, Guangdong province
S3	Zhuwan county, Guangdong province
S4	Nanhuan county, Guangdong province
S5	Gujing county, Guangdong province
S6	Lianhe county, Guangdong province
S7	Gujing county, Guangdong province
S8	Shuangshui county, Guangdong province
S9	Tianbian county, Guangdong province
S10	Dazhe county, Guangdong province
S11	Yamen county, Guangdong province
S12	Chakeng county, Guangdong province
S13	Xinhui city, Guangdong province
S14	Lianhe county, Guangdong province

**Table 2:** UPLC calibration curve data for reference standards.

Compound	Wavelength (nm)	Regression equation	Correlation coefficient (*R*^2^)	Linear ranges (*μ*g/mL)
Hesperidin	283	*Y* = 6453.5*X* − 91994	0.9999	262∼1046
Tangeretin	323	*Y* = 2 × 10^10^*X* − 41461	0.9999	0.0159∼0.080
Nobiletin	330	*Y* = 10^10^*X* − 20835	0.9995	0.048∼0.144
5-Demethylnobiletin	340	*Y* = 10^10^*X* − 36311	0.9999	0.041∼0.247

**Table 3:** The precision, stability, repeatability, and recovery of four references.

Peak	Precision (RSD%)	Stability (RSD%)	Repeatability (RSD%)	Recovery (RSD%)
Hesperidin	0.67	1.80	1.04	2.02
Tangeretin	0.76	0.92	0.88	2.05
Nobiletin	0.51	0.79	0.94	2.14
5-Demethylnobiletin	0.82	0.84	1.29	1.87

**Table 4:** Relative retention time of common peaks in fourteen batches of samples.

Peak	S1	S2	S3	S4	S5	S6	S7	S8	S9	S10	S11	S12	S13	S14	RSD (%)
1	0.24	0.24	0.21	0.21	0.21	0.21	0.20	0.21	0.21	0.21	0.21	0.21	0.21	0.21	5.47
2	0.31	0.30	0.28	0.28	0.28	0.28	0.28	0.28	0.28	0.28	0.28	0.28	0.28	0.28	3.49
3	0.32	0.32	0.29	0.29	0.29	0.29	0.29	0.29	0.29	0.29	0.29	0.29	0.29	0.29	2.99
4	0.36	0.36	0.34	0.33	0.33	0.33	0.33	0.33	0.33	0.33	0.33	0.33	0.33	0.33	2.59
5	0.44	0.44	0.42	0.42	0.42	0.42	0.42	0.42	0.42	0.42	0.42	0.42	0.42	0.42	1.59
6	0.47	0.47	0.46	0.45	0.45	0.45	0.45	0.45	0.45	0.45	0.45	0.45	0.45	0.45	1.53
7	0.51	0.51	0.50	0.50	0.50	0.50	0.50	0.50	0.50	0.50	0.50	0.50	0.50	0.50	1.13
8	0.55	0.55	0.54	0.54	0.54	0.54	0.54	0.54	0.54	0.54	0.54	0.54	0.54	0.54	0.84
9	0.69	0.69	0.69	0.69	0.69	0.69	0.69	0.69	0.69	0.69	0.69	0.69	0.69	0.69	0.31
10	0.72	0.72	0.72	0.72	0.72	0.71	0.72	0.72	0.72	0.72	0.71	0.72	0.72	0.71	0.37
11	0.76	0.76	0.75	0.75	0.75	0.75	0.75	0.75	0.75	0.75	0.75	0.75	0.75	0.75	0.19
12	0.83	0.83	0.83	0.83	0.83	0.83	0.83	0.83	0.83	0.83	0.83	0.83	0.83	0.83	0.17
13	0.90	0.90	0.90	0.90	0.90	0.90	0.90	0.90	0.90	0.90	0.90	0.90	0.90	0.90	0.06
14	0.94	0.94	0.94	0.94	0.94	0.94	0.94	0.94	0.94	0.94	0.94	0.94	0.94	0.94	0.04
15	0.95	0.95	0.95	0.95	0.95	0.95	0.95	0.95	0.95	0.95	0.95	0.95	0.95	0.95	0.04
16	0.97	0.97	0.97	0.97	0.97	0.97	0.97	0.97	0.97	0.97	0.97	0.97	0.97	0.97	0.01
17(s)	1.00	1.00	1.00	1.00	1.00	1.00	1.00	1.00	1.00	1.00	1.00	1.00	1.00	1.00	0.00
18	1.68	1.69	1.69	1.69	1.69	1.69	1.69	1.69	1.69	1.69	1.69	1.69	1.69	1.69	0.14
19	1.71	1.71	1.72	1.72	1.72	1.72	1.72	1.72	1.72	1.72	1.72	1.72	1.72	1.72	0.14
20	1.79	1.79	1.79	1.79	1.79	1.80	1.80	1.79	1.79	1.79	1.80	1.79	1.80	1.80	0.14
21	1.87	1.87	1.88	1.87	1.87	1.88	1.88	1.87	1.88	1.88	1.88	1.88	1.88	1.88	0.14

**Table 5:** Relative peak areas of common peaks in fourteen batches of samples.

Peak	S1	S2	S3	S4	S5	S6	S7	S8	S9	S10	S11	S12	S13	S14	RSD (%)
1	0.93	4.14	9.3	0.41	1.07	0.71	1.08	7.18	27.13	0.31	0.47	1.16	0.36	0.68	184.58
2	2.06	0.98	2.69	0.95	2.43	1.72	2.44	10.73	62.04	0.7	1.24	2.72	0.81	1.71	242.32
3	0.97	0.5	1.06	0.31	1.08	0.7	1.09	5.35	25.83	0.27	0.69	1.13	0.35	0.67	235.62
4	2.53	1.07	2.88	0.94	2.77	1.87	2.9	9.13	71.71	0.69	1.39	3.04	0.88	1.75	251.87
5	2.7	10.43	26.28	1.29	3	2.53	2.9	9.24	83.41	0.95	1.8	3.53	1.01	2.4	202.81
6	1.13	1.85	1.44	1.13	1.36	0.86	1.02	106.41	46.87	1.44	1.14	1.68	1.33	1.49	246.15
7	0.31	0.63	0.45	0.29	0.4	0.23	0.36	21.79	12.52	0.41	0.29	0.38	0.33	0.51	228.79
8	0.55	1.57	0.74	0.53	0.73	0.35	0.81	75.16	15.56	0.87	0.42	0.62	0.47	0.66	282.64
9	0.42	0.28	0.46	0.46	0.56	0.32	0.4	16.61	21.83	0.4	0.5	0.69	0.4	0.95	217.57
10	0.53	0.43	0.45	0.48	0.68	0.36	0.59	23.07	26.26	0.51	0.64	0.78	0.55	1.13	217.35
11	0.49	0.48	0.6	0.29	0.6	0.48	0.73	2.97	14.84	0.26	0.49	0.78	0.42	0.57	223.80
12	0.44	8.73	4.17	0.28	0.49	0.23	0.56	36.99	10.25	0.51	0.3	0.4	0.3	0.51	216.06
13	1.23	14.18	11.6	0.59	1.36	0.88	1.69	23.49	29.75	0.59	0.79	1.49	0.52	1.13	151.58
14	0.95	1.07	1.05	0.93	1.09	0.87	1.1	58.01	36.79	1.09	0.95	1.3	1.1	0.98	226.31
15	0.23	0.2	0.12	0.09	0.18	0.07	0.2	4.82	4.03	0.1	0.15	0.13	0.08	0.26	204.99
16	0.29	0.16	0.15	0.4	0.15	0.37	0.11	46.18	8.99	0.67	0.25	0.38	0.54	0.44	291.39
17(s)	1	1	1	1	1	1	1	1	1	1	1	1	1	1	0.00
18	1.6	3.18	2.52	2.02	2.23	1.06	1.96	201.78	60.06	2.12	1.26	1.73	1.91	1.85	267.27
19	2.16	35.56	23.83	1.76	2.7	1.63	2.72	124.8	75.67	2.9	2.15	1.77	1.78	1.52	183.05
20	0.41	3.26	3.56	0.86	0.41	0.04	0.43	49.98	16.18	0.5	0.42	0.46	0.72	0.27	243.22
21	0.86	13.81	10.03	1.16	1.14	0.61	1.07	113.94	29.95	1.32	0.77	1.17	1.05	1.03	238.29

**Table 6:** Similarities of UPLC fingerprints.

Sample	S1	S2	S3	S4	S5	S6	S7	S8	S9	S10	S11	S12	S13	S14
S1	1.000													
S2	0.813	1.000												
S3	0.995	0.858	1.000											
S4	0.887	0.968	0.92	1.000										
S5	0.996	0.851	0.998	0.912	1.000									
S6	0.992	0.77	0.982	0.859	0.981	1.000								
S7	0.994	0.838	0.994	0.896	0.997	0.983	1.000							
S8	0.491	0.872	0.557	0.812	0.546	0.432	0.515	1.000						
S9	0.982	0.883	0.991	0.951	0.989	0.965	0.98	0.621	1.000					
S10	0.774	0.973	0.822	0.97	0.81	0.738	0.785	0.907	0.868	1.000				
S11	0.971	0.903	0.985	0.962	0.981	0.955	0.972	0.647	0.994	0.889	1.000			
S12	0.993	0.82	0.991	0.895	0.99	0.988	0.991	0.501	0.985	0.788	0.975	1.000		
S13	0.821	0.963	0.863	0.986	0.85	0.795	0.83	0.862	0.905	0.987	0.926	0.836	1.000	
S14	0.963	0.907	0.98	0.962	0.977	0.939	0.965	0.664	0.992	0.892	0.99	0.968	0.922	1.000
*R*	0.979	0.908	0.992	0.961	0.989	0.961	0.982	0.648	0.997	0.884	0.996	0.981	0.917	0.993

**Table 7:** Relative content of four flavonoids.

Sample	Hesperidin (*μ*g/g)	Tangeretin (*μ*g/g)	Nobiletin (*μ*g/g)	5-demethylnobiletin (*μ*g/g)
1	3394.84	0.91	4.45	1.82
2	461.75	0.55	5.31	2.12
3	340.93	0.32	1.75	0.78
4	1079.05	0.54	1.00	0.69
5	2714.44	0.72	4.33	1.89
6	1091.80	0.09	0.93	0.40
7	1140.69	0.32	1.62	0.68
8	261.28	0.98	2.28	2.14
9	303.84	0.83	3.58	1.47
10	829.73	0.26	1.15	0.57
11	2692.53	0.74	3.42	1.28
12	1414.10	0.42	1.37	0.95
13	962.85	0.41	0.86	0.55
14	2073.46	0.39	1.85	1.28

**Table 8:** IC_50_ values.

No	IC_50_ (mg/mL)
L-ascorbic acid	0.061
S1	2.232
S2	2.736
S3	3.15
S4	3.543
S5	2.651
S6	2.822
S7	1.685
S8	4.455
S9	3.317
S10	4.122
S11	5.047
S12	2.872
S13	2.41
S14	1.578

**Table 9:** Eigen values and contribution rate of 14 samples.

Principal components	Initial eigenvalue	Variance contribution rate (%)	Cumulative contribution rate (%)
1	14.565	69.358	69.358
2	2.585	12.308	81.666
3	2.367	11.269	92.936
4	0.497	2.367	95.303
5	0.446	2.125	97.428
6	0.224	1.067	98.495
7	0.154	0.734	99.228
8	0.069	0.326	99.555
9	0.046	0.218	99.773
10	0.031	0.148	99.921
11	0.013	0.063	99.984
12	0.002	0.009	99.993
13	0.002	0.007	100

**Table 10:** Loading matrix analysis results of 21 common peak principal components in 14 samples.

Common peak	Load		
	PC1	PC2	PC3
1	0.876	−0.255	0.325
2	0.929	−0.331	0.032
3	0.937	−0.309	0.053
4	0.925	−0.323	0.056
5	0.894	−0.315	0.255
6	0.926	0.175	−0.317
7	0.953	0.042	−0.237
8	0.804	0.43	−0.284
9	0.883	−0.157	−0.246
10	0.899	−0.133	−0.243
11	0.915	−0.376	−0.026
12	0.527	0.514	0.631
13	0.775	−0.013	0.62
14	0.956	−0.023	−0.236
15	0.937	−0.146	−0.035
16	0.536	0.483	−0.617
17	0.73	−0.387	0.013
18	0.85	0.36	−0.312
19	0.661	0.332	0.635
20	0.705	0.584	−0.05
21	0.647	0.678	0.328

**Table 11:** The results of grey relational coefficient of 14 samples.

Peak no	Correlation coefficient
X6	0.7333
X14	0.7328
X7	0.7306
X13	0.7281
X16	0.7272
X20	0.7091
X17	0.7074
X9	0.7063
X19	0.7022
X10	0.7003
X18	0.6978
X21	0.6970
X11	0.6863
X15	0.6728
X8	0.6663
X12	0.6395
X3	0.6392
X1	0.6328
X5	0.6276
X4	0.6263
X2	0.6256

**Table 12:** The results of dose-effect correlation coefficient.

Peak	Flavonoids	Correlation coefficient	Average contents (*μ*g/g)
20	Tangeretin	0.7365	0.53
21	5-Demethylnobiletin	0.6711	1.19
19	Nobiletin	0.6385	2.42
17	Hesperidin	0.6261	1340.09

## Data Availability

The data used to support the findings of this study are included within the article.
